The article "Short Text Paraphrase Identification Model Based on RDN-MESIM" was published in 2021. Journal: Comput Intell Neurosci.

# Short Text Paraphrase Identification Model Based on RDN-MESIM

**DOI:** 10.1155/2021/6865287

**Published:** 2021-09-05

**Authors:** Jing Li, Dezheng Zhang, Aziguli Wulamu

**Affiliations:** ^1^School of Computer and Communication Engineering, University of Science and Technology Beijing, Beijing 100083, China; ^2^Beijing Key Laboratory of Knowledge Engineering for Materials Science, University of Science and Technology Beijing, Beijing 100083, China

## Abstract

In the rapid development of various technologies at the present stage, representative artificial intelligence technology has developed more prominently. Therefore, it has been widely applied in various social service areas. The application of artificial intelligence technology in tax consultation can optimize the application scenarios and update the application mode, thus further improving the efficiency and quality of tax data inquiry. In this paper, we propose a novel model, named RDN-MESIM, for paraphrase identification tasks in the tax consulting area. The main contribution of this work is designing the RNN-Dense network and modifying the original ESIM to adapt to the RDN structure. The results demonstrate that RDN-MESIM obtained a better performance as compared to other existing relevant models and archived the highest accuracy, of up to 97.63%.

## 1. Introduction

With the rapid development of computer technology and the overall popularization of the Internet, the global digital information storage capacity has been growing explosively. Abundant information resources not only bring convenience to people's life and production but also lead to the problem of information data duplication and redundancy. These text data are sparse, real-time, nonnormative, and other characteristics, resulting in the manual processing of this massive text information which is extremely difficult. The paraphrase identification (PI) for user-generated noisy text is an important task in natural language processing, for example, question answering, semantic disambiguation, text summarization, information extraction, and recommendation systems. Recently, the task of PI has gained widespread attention in natural language processing due to the need to solve the influence of language variation.

PI is a critical task in natural language processing (NLP). PI definition recognition, also known as paraphrase detection, is usually formalized as a binary classification task: for given two sentences, determine if they are in paraphrase relation or not. Sentences with the same meaning are called paraphrase pairs, and sentences with different meanings are called nonparaphrase pairs [1]. It has been considered for determining different linguistic expressions with similar meanings. In other words, they are annotated with the binary classification task: given two sentences (S1 and S2), the result of measuring whether they have the same represented intention will then be defined as 0 or 1 [2]. With the increasingly prominent performance of deep learning in the machine learning research area, deep learning has been widely used in natural language processing, speech recognition, image processing, and other fields. Due to the flexible structure of deep learning, it can abstract local features and have a memory function, which makes deep learning stand out from many algorithms. In natural language processing, deep learning has also shown its powerful advantages.

The article "Short Text Paraphrase Identification Model Based on RDN-MESIM" was published in 2021. Journal: Comput Intell Neurosci.

The underlying artificial intelligence applications that tax intelligence consulting [3] service relies on are of different maturity due to different complexity of use scenarios and different levels of technology development. In the core technology of intelligent consultation, speech recognition and natural language understanding and generation have been relatively mature applications. However, the application maturity of natural language processing and deep learning is relatively low. If there is no breakthrough and innovation in the algorithm and computing power of the existing technology, the improvement of question matching degree and reply accuracy rate is also relatively limited.

In order to solve the above problems, PI, a traditional task in NLP, combined with deep learning, will be applied to the intelligent tax inquiry service. It will simplify the process and procedures of tax collection, increase the efficiency and quality of office work, accelerate the informatization process of tax reform, and provide better services to taxpayers [4].  Figure 1 demonstrates the relationship among deep learning, natural language processing, and tax intelligence consulting service.

In short, this paper mainly contributes to the following aspects:

Propose a novel network structure RDN to implement multiple uses of short text features and a novel model RDN-MESIM for PI task which attains rich semantic information of tax question pair, and the results outperformed other models.

Resolving the tax intelligence consulting question pairs by combining PI tasks: the RDN-MESIM attains features from tweet word and single word levels, and RDN provides the service of integrating these features with multiple using of them, which gives benefit to attain the hierarchical semantic relationship among the tax question pairs.

The rest of the paper is organized as follows: in Section 2, the related work on PI will be presented.  Section 3 presents our proposed novel approach for PI. In Section 4, we will talk about the experiment result. Finally, the conclusion and the future expectations will be introduced in Section 5.

The article "Short Text Paraphrase Identification Model Based on RDN-MESIM" was published in 2021. Journal: Comput Intell Neurosci.

## 2. Related Work

In recent years, researchers have conducted a large amount of research in definition recognition. The existing methods of paraphrase recognition mainly include a feature-based method and a neural network-based method. When compared to the previous work on sentence modelling, most of them have focused on feature engineering to improve the performance of their sentence pair modelling such as *n*-gram overlap features [5], syntax features [6, 7], and linguistic features [8]. For instance, the assessment metrics for machine translation evaluating semantic similarities between two sentences. It is based on word-level or character-level *n*-gram overlapping [9]. In addition to lexical semantics, a syntax-based approach is also proposed [10]. The knowledge-based approach uses WordNet to detect synonyms. Therefore, the systems can identify expressions that have the same meaning in the definition [11].

Recently, deep learning techniques have moved researchers' attention to semantic distributed representations. A variety of deep neural network-based architectures have been proposed. Commonly used Neural Network models include Convolutional Neural Network (CNN), Return Neural Network (RNN), and attention mechanism. On the basis of these models, scholars have put forward various Neural Network models applied to definition recognition.

Through the massive click exposure logs of Query and Document in the search engine, DSSM [12] uses the DNN deep network to express Query and Document as low-dimensional meaning vectors, and the distance between the two semantic vectors is calculated through the cosine similarity, and finally, the semantic similarity model is trained. Then, this model will be applied to predict the similarity of two sentences at the semantic level and then obtain the low-dimensional embedding vector of the sentences. The biggest feature of the DSSM model is that Query and Document are two independent subnetworks. Then, this feature is transplanted to the recall link of the recommendation algorithm, which is the independent tower structure of the subnetwork, built for User and Item, respectively. However, DSSM has the inherent disadvantage of losing contextual information. Then, CDSSM [13] was proposed, and it can make up for the DSSM's disadvantage. Its structure is also very simple, mainly replacing DNN with CNN. Since the purpose is to record the context of the input sentence, LSTM is undoubtedly better at this model, so there is a DSSM model constructed by LSTM which named LSTM-DSSM [14]. MV-DSSM [15] can be generally understood as multiview DSSM. In the original DSSM, two types of embedding, Query and Doc, need to be trained, and the ownership weight of the DNN is shared. However, MV-DSSM can train more than two types of training data, and the parameters of the depth model are independent of each other. DSSM based on multiview has more parameters. Due to the training from multiple perspectives, the input corpus can also be different and the degree of freedom is greater. But the problem is that training becomes more and more difficult.

The article "Short Text Paraphrase Identification Model Based on RDN-MESIM" was published in 2021. Journal: Comput Intell Neurosci.

MVLSTM [16] is a multisemantic model based on the bidirectional LSTM network is proposed. This model can extract the important features of sentences more efficiently and has achieved good results in the experiment. In this paper, two-way LSTM is used to process two sentences, and then, the matching degree is calculated pair by the output of the hidden layer of LSTM. It is a multiview (MV) process, which can examine the meaning of each word in different contexts. Simultaneously, using bidirectional LSTM to process the sentence is equivalent to using a variable length window to interpret the sentence step by step and realize the effect of multigranularity inspection of the sentence.

For the text matching model, Hu et al. [17] put forward two kinds of networks: ARC-I uses CNN characteristics of text extraction and then calculates the similarity of features. However, in this model, when extracting features, there is no interaction between the two texts. In order to solve this problem, the paper extracted the characteristics of each text including considering their interaction, then ARC-II structure was proposed.

ABCNN [18] is mainly designed to solve the sentence correctness problem, based on these three tasks, Answer Selection (AS), Paraphrase Identification (PI), and Textual Entailment (TE). It comes up with that most of the previous models are fine-tuning sentences in specific tasks or generating semantic representations for each sentence independently, as well as using linguistic methods that have not taken into account the interdependent information between sentences. In the basic BiCNN, two parallel CNN layers are constructed to extract features of sentences, respectively, and convolution parameters are shared between the two layers, followed by conventional operations such as pool. Finally, a Logistic Regression is used for classification. Then, attention-based BCNN has three parts: ABCNN-1, ABCNN-2, and ABCNN-3. The basic idea of ABCNN-1 [18] is to generate an attention matrix A according to the feature map of two sentences before convolution and then perform matrix multiplication of matrix *A* and parameter *W*. A new attention feature map with the same size as the original feature map is constructed as another channel of convolution input, and then, convolutional pooling and other operations are carried out. It is hoped that the attention feature map can play a feature of extraction with concerns during convolution operation. Compared with ABCNN-1, which conducts attention operation before convolution, and ABCNN-2 [18], which conducts attention operation before the pooling layer, the construction of the attention matrix is consistent with ABCNN-1, but the convolution output is reweighted before pooling. The attention of ABCNN-2 works at higher dimensions. Attention before the convolution layer works at the word level. Attention before the pooling layer works at the phrase level. At the same time, compared with ABCNN-1, ABCNN-2 requires less computation and has no parameter *W*, so it is stronger in resisting overfitting. Combining the advantages of ABCNN-1 and ABCNN-2, the author proposes ABCNN-3 [18], which combines the two models.

The article "Short Text Paraphrase Identification Model Based on RDN-MESIM" was published in 2021. Journal: Comput Intell Neurosci.

ESIM [19] is a model that integrates BiLSTM and attention mechanism. It is to send the input sentence to the BiLSTM network by word embedding or directly using pretrained word vectors and to perform attention calculation on the output of the LSTM network; then, the difference will be calculated. The two difference matrices are fed into the BiLSTM network again, and the output of the LSTM network is averaged and maximum pooling. Finally, the pooling output is fed into the multilayer perceptron classifier, and SoftMax is used for classification. In conclusion, it has fine design sequential inference structures and considers local inference and global inference. ESIM has been pursuing the use of BiLSTM to obtain the representation of the context information of the sentence, but has neglected the representation of the sentence itself to some extent.

DenseNet [20] is a connected convolutional network which constructs the connection relationship between different layers, makes full use of feature, and further reduces the gradient disappeared problem. Besides, it utilizes bottleneck layer, translation layer, and smaller growth rate to make the network become narrow and parameters become less, which effectively restrain the overfitting and also reduce the amount of calculation. DenseNet is transformed from resnet [21], but it does not use the traditional residual link. It applies the concatenate method to link each layer output and then inputs them into the following layer. In other words, each layer will receive the information that comes from the former layer. The structure of the DIIN [22] model is similar to that of other matching models, and CNN and LSTM are also used for feature extraction. However, in its input layer, the author puts forward many ideas, including word vector, and adds some additional features such as part of speech. The intention is to input some additional syntactic features. The CNN part also adopts the structure of DenseNet [20]. Scholars such as Kim et al. [23], inspired by the DenseNet, compared the RNN Dense link, combined the attention mechanism, and designed the DRCN model. However, with the depth of network deepening, data dimension will become bigger, which will be easy to cause OOM. According to the above problem, the author adopts the autoencoder as the bottleneck of data dimension reduction.

The article "Short Text Paraphrase Identification Model Based on RDN-MESIM" was published in 2021. Journal: Comput Intell Neurosci.

## 3. Methodology

In this section, the proposed approach for tax consulting questions' PI task is discussed in detail.  Figure 2 depicts the proposed framework, and details are presented in subsequent sections.

### 3.1. Data Preprocessing

The dataset used in this experiment is collected from our project. There are totally 54716 question pairs. A subset of the dataset has been used to train the neural network (43419 question pairs: 79% training dataset), and the other part of the data (11297 question pairs: 21%) was used to test and validate the performance of the trained neural network. The amount of the test dataset is 8693 question pairs, and the validation dataset is 2604 question pairs. There were two types of label in the dataset: 0 and 1. 0 represents that the two questions express different meanings, while 1 demonstrates that the two questions have similar meaning. Totally, there are 27410 question pairs and 27306 question pairs in the whole dataset, which have 1 and 0 labels, respectively. In the training dataset, test dataset, and validation dataset, there are three table headers: sentence1, sentence2, and label. Every piece of data contains question 1, question 2, and 0/1, separated by commas.

After the step of data collection, the dataset has been preprocessed using tokenization and normalization. In order to tokenize question pairs, the jieba tokenizer is used. For example, “如何确定个税法中的纳税年度 (how to determine the pay tax year in individual income tax)” is tokenized into “如何(how),” “确定(determine),” “个税法 (individual income tax),” “中 (prepositions),” “的 (prepositions),” “纳税 (pay tax),” and “年度 (year).” The normalization technique is used to replace punctuation and stop words such as “呢 (modal particle),” “吗 (modal particle),” and “哦 (modal particle).” Figure 3 shows examples of question pairs.

### 3.2. RNN-DenseNet (RDN)

Tax intelligence consulting questions have not too long word lengths compared to community questions and are relatively more informative. According to the feature of the dataset, we chose ESIM as the fundamental method, which has high speed of training procedure. ESIM uses only BiLSTM to learn to represent a word and its context in the encoding layer, and we think it is an area to enrich the representation layer of it, and then, we add the feature extraction method and modified it to adapt to our PI task and repeated trials to assure the availability of the proposed architecture.

The article "Short Text Paraphrase Identification Model Based on RDN-MESIM" was published in 2021. Journal: Comput Intell Neurosci.

As we know, DenseNet [20] is transformed from resnet [21], and it reuses features directly by making dense connections between all the previous layers. Inspired by DIIN [22], we applied this RDN structure into our model.  Figure 4 shows the whole of the RDN structure. As information shown in Figure 4, two parts are included which are dense block and transition layer. The number of the dense block and transition layer pairs is decided by our experiments' result which will be explained in Section 4. Dense block defines how the inputs and outputs are connected, and the transition layer controls the number of channels so that it is not too large.

In every dense block, five parts have been designed: BiLSTM layer, L2 normalization, soft-attention [24] layer, concatenate layer, and batch normalization. In fact, the attention mechanism has been widely used in many fields in computer vision (such as classification, detection, segmentation, model generation, and video processing), and these works have also derived many different attention methods. The common part of these methods is to use the relevant features to learn the weight distribution and then apply the learned weight to the features to further extract the relevant knowledge, but the way weights are applied is slightly different. In our experiment, we apply attention to the channel of the data characteristics. After the calculation from the BiLSTM layer and L2 normalization layer, the attention layer will learn the weight form every dimension. Then, the output from the original embedding, BiLSTM and L2 normalization, and attention will be concatenated together to feed into batch normalization to wait for inputting into the transition layer.

Figure 5 demonstrates the structure of dense block. A step-by-step explanation of the dense block in RDN is described below: given two question sentences' pairs {*Q*_1_, *Q*_2_} which contain *m* and *n* words, respectively, their embeddings *X*_question1_ = {*x*_1_, *x*_2_,…, *x*_*m*_} and *X*_question2_ = {*x*_1_, *x*_2_,…, *x*_*n*_} are sequentially fed in BiLSTM, *X*_question *i*_ is the input of LSTM at time step *i*, $\overset{⟶}{L}$ is the forward LSTM, $\overset{\leftarrow }{L}$ is the backward LSTM, and the encoding process is

(1) $$\begin{array}{c} \overset{⟶}{h_{i}}=\overset{⟶}{L}\left(X_{\text{question }i},\overset{⟶}{h_{i-1}}\right),\\ \overset{\leftarrow }{h_{i}}=\overset{\leftarrow }{L}\left(X_{\text{question }i},\overset{\leftarrow }{h_{i+1}}\right),\\ h_{i}=\left[\overset{⟶}{h_{i}},\overset{\leftarrow }{h_{i}}\right],\\ C\left(X_{\text{question}}\right)=\left[h_{1},h_{2},\ldots ,h_{l}\right], \end{array}$$

where $\overset{⟶}{h_{i}}$ is the hidden state of $\overset{⟶}{L}$ at time step *i*, $\overset{\leftarrow }{h_{i}}$ is the hidden state of $\overset{\leftarrow }{L}$ at time step *i*, and *C*(*X*_question_) is the output which will then be calculated by the L2 normalization layer. From the encoding process, *C*(*X*_question_)_*l*2 normalized_ represents the output of L2 normalization with the input of *C*(*X*_question_), *w*_*α*_^*T*^ is the parameter that can be trained; then, the added attention can be calculated as

(2) $$\begin{array}{c} A_{ij}=w_{\alpha }^{T}C{\left(X_{\text{question}}\right)}_{l2\text{ normalized}},\\ a\left(h_{i}\right)=\sum_{i=1}^{k}\frac{\exp\left(A_{ij}\right)}{\sum_{b=1}^{k}A_{bj}}h_{j},\\ A\left(w\right)=\left[a\left(h_{1}\right),a\left(h_{2}\right),\ldots ,a\left(h_{l}\right)\right], \end{array}$$

where *A*(*w*) is the output of the attention. From the former procedure, *X*_question1_, *X*_question2_, *C*(*X*_question_), and *A*(*w*) have already been calculated; then, the output of the concatenate layer is

(3) $$\begin{array}{c} V_{\text{question}1}=\text{concatenate}\left(X_{\text{question}1},C\left(X_{\text{question}}\right),A\left(w\right)\right),\\ V_{\text{question}2}=\text{concatenate}\left(X_{\text{question}2},C\left(X_{\text{question}}\right),A\left(w\right)\right). \end{array}$$

Then, the output *V* will be applied batch normalization to produce the output of the dense block. In every transition layer, dense layer and batch normalization will be applied to calculate the output.

The article "Short Text Paraphrase Identification Model Based on RDN-MESIM" was published in 2021. Journal: Comput Intell Neurosci.

### 3.3. RNN-MESIM

ESIM [19] model is mainly used for text reasoning. Given a premise *p*, hypothesis *h* is derived, and the goal of its loss function is to determine whether *p* and *h* are related and whether *h* can be deduced from *p*. Therefore, the model can also do text interpretation recognition. The objective of the loss function is to determine whether the two sequences are synonymous sentences, and its structure is shown in Figure 2, which consists of the embedding layer, encoding layer, local recognition layer, recognition composition layer, and decision layer.

The main role of the embedding layer is to map the questions to a vector space and transform it to vector as presentation. The main procedure is we begin to experiment with tweet word and single-word vector training to obtain a trained model for all text by Word2Vec afterword segmentation on all question pairs which are shown in Figure 3. For processing the question pairs' text, we generate a vocabulary for them, count the frequency of each word, and sort the most frequent *V* words from high to low. We select skip-gram combined hierarchical SoftMax as our training model which we have to assure the window size to generate the training samples for our tweet word and a single word. The core content of hierarchical SoftMax is the Huffman tree. Symbols with higher occurrence probability use shorter encoding, while symbols with lower occurrence probability use longer encoding. Then, we get two kinds of vector representation of each sentence which will then be concatenated to calculate sentence representation based on tweet word and a single word in a certain question sentence.  Figure 6 shows the process of calculating sentence representation.

In RDN-MESIM, after attaining the sentence representation from Figure 6, they will be fed into the BiLSTM network which is located at the beginning of the encoding layer in RDN-MESIM to do feature extraction which has been constructed by time sequence and including context information. Our RDN structure will then be applied to do multiple uses of feature. Until now, our encoding layer of our model has been finished; then, data will be fed into our local recognition layer which mainly consists of the attention mechanism. After that, the recognition composition layer will start to work. The second BiLSTM layer has been applied to produce the input for the next layer. The main formulas for this layer have a resemblance to the first BiLSTM; thus, we omit some details of it. The feature has been emphasized again after attention weight is implemented in this layer. The output of this layer has been fed into three layers, respectively. They are average pooling layer, max pooling layer, and *k*-max pooling layer. Then, three parts of the output have been inputted into the concatenate layer to produce the final vector. Finally, score calculation is performed by the RDN-MESIM prediction layer. Our prediction layer in our RDN-MESIM model includes a multilayer perceptron which consists of a hidden layer with the ReLU activation function and SoftMax as the output layer.

## 4. Experiments and Results

In this section, we describe the experimental setup, followed by result and discussions. To assess the performance of our proposed approach, the tax intelligence consulting question pairs' data has been used. The processing process of the data has been described in Section 3.

The article "Short Text Paraphrase Identification Model Based on RDN-MESIM" was published in 2021. Journal: Comput Intell Neurosci.

### 4.1. Experimental Configuration

The system used in this experiment is Ubuntu 20.04.2 LTS, the programming language is python3.7, the deep learning framework is TensorFlow, the graphics card is one Nvidia GeForce RTX 3070 with 8G memory, and CUDA version is 11.0. The optimizer selected is Adam. For testing with the model, the parameters of them are as follows: word embedding dimensions are 200, number of epochs equals to 50, and batch size is 128. For the training process, we set the early stopping method to save time for each model.

### 4.2. Evaluation Criterion

In Table 1, trainable parameters of the models or other modified networks have already been listed. In addition, to assess the performance of proposed approaches, Tables 2 and 3 show the accuracy results by several contrast experiments and Tables 1 and 4 show both loss and accuracy results. The prediction accuracy, precision, recall, *F*_measure_ are used as performance matrices:

(4) $$\begin{array}{c} \text{accuracy}=\frac{\text{TP}+\text{TN}}{\text{TP}+\text{TN}+\text{FP}+\text{FN}},\\ \text{precision}=\frac{\text{TP}}{\text{TP}+\text{FP}},\\ \text{recall}=\frac{\text{TP}}{\text{TP}+\text{FN}},\\ F_{\text{measure}}=2*\frac{\text{precision}*\text{recall}}{\text{precision}+\text{recall}}, \end{array}$$

where TP, TN, FP, and FN represent true positive, true negative, false positive, and false negative, respectively.

### 4.3. Experiment Results

Table 2 presents the results of our proposed RDN-MESIM compared to other existing models where the best performance on the tax question pairs is highlighted in boldface. All parameters in each model have been set based on their original setting, and they have been fine-tuned into better performance on our tax question pairs' data. The results show that RDN-MESIM outperformed other models. Our model attains the best performance with a precision, recall, and *F*_measure_ of 0.9889, 0.9612, and 0.9748, respectively, and an accuracy of 97.63%.

Table 3 indicates the results for ESIM when it is combined with our proposed RDN structure in its different layers. These three layers are Encoding Layer (EL), Local Inference Layer (LIL), and Inference Composition Layer (ICL). The dense block and transition layer pair size are set into 2, which will be modified in the following table. The experiments' results show that the model achieved better performance when our RDN structure is only added into EL of ESIM as compared to other positions of ESIM. It means that this kind of combination way has less trainable parameters and uses less time to train the model and produce the best result.

Table 1 presents the comparison results for different sizes of dense block and transition layer pairs in RDN. The whole contrast experiments are conducted based on adding RDN into EL of ESIM. The reason is that the performance of this condition is the best compared to other situations. Additionally, the results for two pairs of dense block and transition layer outperformed other architectures compared with 3-, 4-, 5-, and 6-pairs' structure.

The article "Short Text Paraphrase Identification Model Based on RDN-MESIM" was published in 2021. Journal: Comput Intell Neurosci.

Table 4 presents the comparison results of the original ESIM combining the traditional deep learning method. The results show that traditional deep learning methods, such as BiGRU [26], can improve the performance of original ESIM to some extent. However, results also prove that our proposed model RDN-MESIM outperformed these methods.

According to the experimental results, our proposed RDN-MSIM model outperformed all other methods. In addition, it is observed that BiGRU [26], CNN can effectively judge the similarity of the question pairs. With the improved model based on ESIM, we achieve excellent results by combining the proposed RDN network structure and modify the original ESIM to do more feature extraction and apply them to the model. Analyzing the reasons, the existence of ESIM is to inference the premise and hypothesis, and it lacks more useful features to finish the tasks, especially when it comes to PI tasks. Thus, our RDN is the neural network that has an obvious advantage in feature extraction and multiple uses. The other modification of the original ESIM has also improved the characteristic utilization. The experiments prove that our novel network RDN-MESIM archives excellent results in PI tasks in the tax intelligence consulting area.

## 5. Discussion

In this paper, we proposed a novel structure that combines tweet word and single word semantic information and multiple uses them to PI task on tax question pairs' data. According to the results in Table 2, our approach greatly outperforms the other baselines. The ARCII [17] *F*_measure_ is a strong baseline and performs best out of the comparison methods. It mainly uses 1D Convolution to encode the embedding and then performs matching calculation. Although it has a procedure to process the simplex level of semantic information and attain a nice result, our model is better in performance with considering the interaction of the text information in the following local recognition layer and the multiple uses of features. This shows the importance of local semantic features in the PI task on tax question pairs.

The position of the multiple utilization feature has a significant influence on our model performance. From the results in Table 3, we observe that RDN gives a positive influence when it is combined in the encoding layer rather than other layers. This proves that the feature utilize should be processed well before the interaction or other operation calculation. The combined feature has rich semantic information, and it has been utilized in a suitable time which has been proved in Figure 3.

The article "Short Text Paraphrase Identification Model Based on RDN-MESIM" was published in 2021. Journal: Comput Intell Neurosci.

The comparison experiments shown in Figure 4 illustrate that our model improves the task performance greatly. From the table, we can conclude that the CNN combing attention mechanism and L2 normalization produce a better result with a precision, recall, *F*_measure_, and loss of 0.9796, 0.9542, 0.9667, and 0.0945, respectively, and an accuracy of 96.99%. For our RDN network, we mainly use BiLSTM and attention in the dense block to cooperate with composition layer. BiLSTM contains time extension neurons with multiple time outputs which are calculated, and it can be used to describe the output of a continuous state in time. In other words, BiLSTM has a nature advantage to process text compared to CNN. Therefore, compared with the other network, this design is explainable and purposeful.

The limitation of our model is the semantic information is not enough for tax question PI task since there are more professional words in the question data. In order to represent them in a better compound mode, the following progress of our project will be considering adding external knowledge or applying the pretraining language model to enrich the representation ability of our model and produce better results. Then, we plan to conduct additional research on this challenge.

## 6. Conclusions

Tax intelligence consulting is a complicated process, which requires more information to be demonstrated clearly; however, almost all of the relevant question are short and contain many professional terms. Therefore, the feature of the question should be described at a different level to capture the information of the questions to the greatest extent. Our model greatly improves the accuracy of PI tasks in the tax intelligence consulting area. The reasons can be concluded: RDN-MESIM has the advantage of representing question pairs in different levels and does multiple uses of features. Through modifying the structure of original ESIM to adapt to our tax questions, combining the inference ability to attain the sentence logical relationship helps our PI task to some extent. The LSTM layer plays a certain role in our model, and its application field is extremely wide. It can not only be applied to the tax field mentioned in the paper but also can be applied to predicting the stability of a smart grid [27]. In addition to LSTM, CNN is another structure that we will explore and apply to the tax field next. Although it is mostly applied to the image field, such as predict diabetic retinopathy [28], it is still popular in text-related fields. The future work for feature engineering will be combining external knowledge or pretraining the language model to strengthen the model's robust ability and also explore more features such as linguistic relationships [29] to improve the model ability to another level.

The article "Short Text Paraphrase Identification Model Based on RDN-MESIM" was published in 2021. Journal: Comput Intell Neurosci.

## Figures and Tables

**Figure 1:** Relationship among deep learning, natural language processing, and tax intelligence consulting service.

**Figure 2:** Proposed RDN-MESIM framework.

**Figure 3:** Tax question pairs' example.

**Figure 4:** Proposed RDN structure.

**Figure 5:** Proposed dense block structure of RDN.

**Figure 6:** Sentence representation processing.

**Table 1:** The results in different depths of RDN's dense block and transition layer pair.

Layer	Loss	Accuracy	Trainable parameter
2	0.0956	0.9710	1,933,570
3	0.1363	0.9615	3,257,602
4	0.1271	0.9610	4,977,922
5	0.1351	0.9638	7,094,530
6	0.1768	0.9412	9,607,426

**Table 2:** Different models results on PI task using tax intelligence consulting question pairs' data.

Model	Precision	Recall	*F*_measure_	Accuracy (%)
DSSM [12]	0.8412	0.8187	0.8297	83.64
CDSSM [13]	0.9380	0.8814	0.9088	92.20
MVLSTM [16]	0.9940	0.9112	0.9508	95.94
ARCII [17]	0.9710	0.9463	0.9584	96.47
ABCNN [18]	0.9559	0.9344	0.9450	94.46
DIIN [22]	0.9763	0.9511	0.9635	96.10
DRCN [23]	0.9401	0.9079	0.9237	93.40
**RDN-MESIM**	0.9889	0.9612	0.9748	**97.63**

**Table 3:** Different position of MESIM applied our proposed RDN structure results on PI task using tax intelligence consulting question pairs' data.

Position	Precision	Recall	*F*_measure_	Accuracy
EL	0.9898	0.9428	0.9639	0.9710
LIL	0.9883	0.9197	0.9527	0.9588
ICL	0.8147	0.7960	0.8052	0.8079
EL + LIL	0.9514	0.9353	0.9432	0.9475
EL + ICL	0.9575	0.9144	0.9354	0.9447
LIL + ICL	0.9810	0.9047	0.9413	0.9473
EL + LIL + ICL	0.5800	0.5217	0.5493	0.5685

**Table 4:** The results of different networks on PI task using tax intelligence consulting question pairs' data based on original ESIM.

Structure	Precision	Recall	*F*_measure_	Loss	Accuracy
ESIM [19]	0.9666	0.9577	0.9621	0.1036	0.9649
+BiGRU	0.9739	0.9310	0.9519	0.1037	0.9610
+BiGRU + Dense + L2	0.9700	0.9311	0.9501	0.1327	0.9575
+BiGRU + CNN	0.9939	0.9505	0.9717	0.0993	0.9738
+K-Maxpooling + Dense	0.9811	0.9404	0.9603	0.1121	0.9689
+CNN + K-Maxpooling + Dense + L2	0.9807	0.9414	0.9606	0.1111	0.9666
+CNN + attention + L2	0.9796	0.9542	0.9667	0.0945	0.9699
+Xception [25]	0.9896	0.9453	0.9669	0.1104	0.9689
**RDN-MESIM**	0.9889	0.9612	0.9748	0.0808	**0.9763**

## Data Availability

The data used to support the findings of the study are available from the corresponding author upon request.
